This article has been retracted.

# An Automatic Web Service Composition Framework Using QoS-Based Web Service Ranking Algorithm

**DOI:** 10.1155/2015/207174

**Published:** 2015-10-01

**Authors:** Deivamani Mallayya, Baskaran Ramachandran, Suganya Viswanathan

**Affiliations:** Department of Computer Science and Engineering, College of Engineering, Guindy, Anna University, Chennai 600025, India

## Abstract

Web service has become the technology of choice for service oriented computing to meet the interoperability demands in web applications. In the Internet era, the exponential addition of web services nominates the “quality of service” as essential parameter in discriminating the web services. In this paper, a user preference based web service ranking (UPWSR) algorithm is proposed to rank web services based on user preferences and QoS aspect of the web service. When the user's request cannot be fulfilled by a single atomic service, several existing services should be composed and delivered as a composition. The proposed framework allows the user to specify the local and global constraints for composite web services which improves flexibility. UPWSR algorithm identifies best fit services for each task in the user request and, by choosing the number of candidate services for each task, reduces the time to generate the composition plans. To tackle the problem of web service composition, QoS aware automatic web service composition (QAWSC) algorithm proposed in this paper is based on the QoS aspects of the web services and user preferences. The proposed framework allows user to provide feedback about the composite service which improves the reputation of the services.

## 1. Introduction

In recent years, the software industry has been dominated by the web services. Most of the enterprises publish their applications on the World Wide Web using web services. Web service technology is the heart of Service Oriented Architecture (SOA) that meets the interoperability demands of the web application. W3C defines web service as “a software system designed to support interoperable machine to machine interaction over a network.” Web services [1] are self-contained, self-describing, and loosely coupled software applications that can be published, located, and accessed across the web using XML-based open standards, namely, SOAP (Simple Object Access Protocol), WSDL (Web Service Description Language), and UDDI (Universal Description, Discovery and Integration).

The three main components in web service architecture are web service provider, web service requester, and UDDI registry [2] as given in Figure 1. The web service provider publishes information about the web services in UDDI registry in the form of WSDL file. WSDL of a web service is a machine-readable description that indicates the service invocation parameters of the web service. WSDL is an XML-based language that describes the functionality of the web service like location of the service and operations (or methods) of the service. Universal Description, Discovery and Integration (UDDI) is a platform-independent, Extensible Markup Language- (XML-) based registry for businesses worldwide to list themselves on the Internet, used to register and locate web service applications. Web service consumer uses UDDI to discover appropriate services which meet the requirement using the service invocation parameters provided by the web service provider.

Research on web services includes web services description discovery, selection, ranking, composition, deployment, execution, monitoring, and adaptation. Web service description deals with specifying all the information required to access and invoke a web service. Web service discovery is the process of locating and gaining access to a web service which satisfy the customer requirements. Web service selection and ranking are to identify best web services which satisfy the user's requirement. Web service composition involves combining a set of compatible atomic web services in order to satisfy the user's requirement, when a single atomic web service could not satisfy the user's requirement. This paper mainly focuses on web service selection, ranking, and composition from the aspect of quality of service (QoS).

Some of the major challenges in web service composition framework are as follows:

- How to select the best web service when there are many available web services of similar functionality.
- What the factors that influence web service selection are.
- How to meet the various requirements of the user.
- How to compose multiple web services automatically when the user's request is not satisfied with a single web service.

QoS of the web service is used to distinguish the functionally similar web services. The proposed framework solves the first challenge by considering QoS for web service selection. The main QoS properties that influence web service selection are execution cost, availability, average response time, successful execution rate, frequency, and reputation. User preferences over these QoS properties play a vital role while ranking the web services. Our automatic web service composition (QAWSC) algorithm meets the local and global constraints specified by the user. The proposed framework generates composition plans automatically when the user's request is not satisfied with a single atomic service. It assigns atomic web service automatically to each task in the user request. Our algorithm also meets multiple QoS requirements specified by the user.

QoS parameters of web services act as a discriminator in identifying the suitable web services from the set of available web services. After the preliminary filtering with respect to the QoS, the web services are ranked based on the user preference (platinum, gold, and bronze, platinum being the highest preference level and bronze being the lowest preference level). The filtering based on the user preference delivers the expected set of web services with respect to the user.

This paper is organized as follows: Section 2 presents an overview of web service selection and composition approaches.  Section 3 describes the QoS metrics used in this paper.  Section 4 explains the proposed web service composition framework.  Section 5 presents the testing environment and our experimental results. We conclude our work in Section 6.

## 2. Related Works

Some of the current approaches for composition first rank the web services before selection. But the performance of this approach is less when compared to composition approaches that does ranking followed by selection. In [3], QoS-based web service selection model is discussed. This method is based on weightage and normalization of functionally similar services. Though this method gets the client's weightage, there is a large difference between the QoS values of a group of functionally similar services and QoS value of another functionally similar service. During normalization the difference between the normalized QoS values becomes negligible. Thus user's weightage does not influence the QoS values while ranking the web services.

Other normalization approach [4] used for web service selection considers only QoS of the services without users QoS requirements and preferences on QoS aspects. But this approach handles the situation when there is no feasible solution to fulfill QoS constraints set by users. QoS-based web service selection method proposed in [5] requires a lot of interactions with users and does not consider user preferences on various concerned QoS aspects.

Web service composition [6] approaches can be classified into manual composition or static composition, semiautomatic service composition and automated web service composition. In manual composition, composition is achieved programmatically through orchestration languages like Web Services Business Process Execution Language (WS-BPEL). Manual composition of services consumes a lot of time and it cannot adapt to the dynamic environment. Semiautomatic service composition involves the end user in the management of composition through a graphical interface, for example, YAHOO PIPES. This kind of approach also requires users with knowledge in the development and consumes a lot of time.

In automatic web service composition, the system processes the user's request and generates the composite service. This paper focuses on automatic web service composition considering functional and nonfunctional aspect of web services. Advantages of using automatic web service composition approach are that it

- minimizes user intervention,
- accelerates the process of producing a composite service that satisfies the user request,
- eliminates the human errors,
- reduces cost.

Four distinct approaches for automated web service composition are workflow based, model-based, mathematics-based, and AI planning approaches. Some of the other approaches include heuristic approaches which use algorithms like genetic algorithm.

Many automatic approaches do not take QoS attributes into account. Gu et al. [7] proposed an approach without considering QoS aspects and it lacks correctness in composition. The workflow approach proposed by Ardagna et al. [8] focused on adaptation and flexibility of service composition modeled as business processes. BPEL process is created and then annotated with global and local constraints. The QoS constraints are expressed in the Service Level Agreement (SLA). WSQosX proposed in [9] is a workflow engine which calculates an execution plan that maximizes the overall QoS. The main limitation is that many candidate web services for the composition are selected which reduces the efficiency of the approach. Workflows are limited to simple schemas and some of the approaches are manual.

Model-based approaches include [10, 11]. The model-based approach proposed in [12] uses UML activity diagrams to model service compositions. The UML diagrams are then used to generate executable BPEL processes using XSLT transformations. Model-based approaches are time-consuming and not fully automated.

Some of the mathematics-based approaches are [13–15]. The QoS aware service composition problem has been defined as mathematical problems such as integer linear planning, single objective problem with QoS constraints, and the multiple objective problem with QoS constraints which are the most common ones. For the service composition, LIP can help to get the best solution without constructing all the possible composite services. However, it can only be available for the composition problems with small volumes since the traditional branch and bound technique has its computation limitations. On the other hand, it also asks for the linearization of the objective function and the corresponding constraints.

The AI based approach proposed in [16] is complex and some of the other approaches based on “AI planning” will not endure when any one of the web service within the composition plan fails.

PSR system (precomputing solutions for web service composition in an RDBMS) proposed by Lee et al. [2] implemented web service composition using a relational database. This approach is efficient in a large number of services, but it does not consider QoS aspects of composition.

These shortcomings motivated us to build QoS aware automatic web service composition framework using a relational database. Our proposed framework is flexible in supporting user preferences over QoS criteria and also allows user to specify the constraints.

## 3. QoS Model

This section explains the QoS properties considered in the proposed work and explains the notations used in this paper.

### 3.1. Preliminary

**Definition 1 .**

A web service is a tuple WS_*i*_(ID, *I*, *O*, ST, *Q*_*s*_), where

(i) ID is the service identifier,
(ii) *I* is a set of input parameters for WS_*i*_,
(iii) *O* is a set of output parameters for WS_*i*_,
(iv) ST denotes the service type,
(v) *Q*_*s*_ denotes the quality-of-service values for WS_*i*_.

**Definition 2 .**

QoS value of web service WS_*i*_ is a tuple *Q*_*s*_(*q*_1_, *q*_2_,…, *q*_*n*_), 0.0 ≤ *q*_*i*_ ≤ 10.0.

(i) *q*_*i*_ denotes the execution cost, availability, frequency, reputation, average response time, and successful execution rate of a WS, where *i* denotes QoS property.

**Definition 3 .**

A composition plan is a tuple CP  (WS_*i*_,…, WS_*n*_, QV_*s*_), where

(i) WS_*i*_ denotes set of atomic services, where *i* ranges from 1 to *n* and *n* denotes the number of tasks,
(ii) QV_*s*_ is aggregated QoS values of CP.

### 3.2. Quality-of-Service Criteria

Quality of service (QoS) of a web service can be used as a discriminating factor that differentiates the functionally similar web service. QoS of a web service [1] can be considered as a set of nonfunctional attributes of the entities used in the path of the web service to the client that bear on the web service ability to satisfy stated or implied needs in an end-to-end fashion. The values of QoS attributes can vary without impacting the core function of the web service which remains constant most of the time during the web service lifetime. If a web service is advertised to have certain values (or range of values) in these QoS attributes, then that web service conforms to provide a certain QoS level.

QoS attributes are classified into domain independent and domain dependent attributes. Attributes like availability and successful execution rate are domain independent attributes. An attribute like the cost is a domain dependent attribute. QoS attributes can be distinguished into measurable and immeasurable ones. A measurable QoS attribute can be measured with the help of one or more QoS metrics. A QoS metric is a concept that encompasses all measurement details for a QoS attribute. They have specific value type and their values are associated with a specific unit. For example, for average execution time, the successful execution rate is measurable. Unmeasurable quality attributes cannot be measured at all. They represent static information which is qualitative in nature. These attributes have specific value type and are unitless. Some QoS attributes [16] that influence the performance of a web service are successful execution rate, availability, service execution cost, average response time, frequency, reputation, and so forth which are explained in Table 1.

*Execution Cost*. The Cost *C*_*ij*_ is the amount that a service requester needs to pay to execute service *S*_*i*_ that implements the task *t*_*j*_. Service provider defines the cost for the service. *q*_*c*_ is denoted as *C*_*ij*_ where *i* denotes the service and *j* denotes the task.

*Average Response Time*. The average response time *q*_*t*_ denoted as *t*_*ij*_ is defined as the average elapse time between the request and response time of a web service *S*_*i*_:

(1) average  response  time qt=∑response  time ti−request  time titotal  number  of  service  trials.

*Availability*. The availability *q*_*a*_ of a web service which is denoted as *A*_*ij*_ is the probability that the service *S*_*i*_ that implements the task *t*_*j*_ can be accessed and used. It is a function of the number of times the service responds to a request and of the number of total requests made to the service.

*Reputation*. The reputation *q*_*r*_ of a web service denoted as *R*_*ij*_ is the measure of its trustworthiness. It depends on the user's experience using the service. Different end users can have different opinions about the same service. Reputation can be defined as the average ranking given to the service by end users:

(2) $$\begin{array}{c} \text{reputation }\left(\;q_{r}\;\right)=\frac{\sum_{i=1}^{n}\text{Rep}\left({\text{WS}}_{i}\right)}{\text{total number of service trials }\left(n\right)}, \end{array}$$

where Rep is accumulated score of reputation.

Users provide feedback about the service and rate the service in the range 1 to 5, where 5 indicates the highest score for the web service.

*Frequency*. The frequency *q*_*f*_ of a web service denoted as *F*_*ij*_ is defined as number of times the clients have used web service *S*_*i*_ that implements the task *t*_*j*_.

*Successful Execution Rate*. Successful execution rate *q*_sr⁡_ of a web service denoted as SR_*ij*_ is the percentage that service requests are responded to. It is calculated as the number of successful executions divided by the total number of service trials:

(3) successful  execution  rate qsr⁡=number  of  successful  executionstotal  number  of  service  trials,

where number of successful executions is success count and total number of service trials is success count + failure count.

### 3.3. Quality-of-Service Aggregated Functions

In the proposed framework, composition plan (CP) has a serial execution pattern and we aggregate the QoS values of atomic services WS_*i*_ in CP using the aggregation functions defined in Table 1.

## 4. Proposed Framework

In this section, we present the user preference based web service ranking (UPWSR) algorithm and automatic web service composition (AWSC) algorithm. We formulate the web service composition problem and describe the core components in automatic web service composition framework. A travel reservation scenario is used to explain the proposed framework.

### 4.1. Problem Definition

Given a user request UR(*T*, QWV, *C*), we need to find the best composite services among the list of services that satisfies the user request where

(i) *T* denotes a set of independent tasks *t*_*i*_, where *i* ranges from 1 to *n* and *n* denotes the number of tasks,
(ii) QWV is QoS weight vector which contains user preferences over QoS criteria:
  (4) $$\begin{array}{c} \text{QWV}=\langle \;{qw}_{1},{qw}_{2},{qw}_{3},\ldots ,{qw}_{6}\;\rangle , \end{array}$$
(iii) *C* denotes the constraint specified by the user.

For example, a travel reservation scenario which is a typical web service composition problem as shown in Figure 2 offers travel, accommodation, and local transport rental services to the customers. The user request consists of a set of tasks like booking flight ticket, reserving hotel rooms, and renting a cab. Atomic services like flight service, hotel service, and taxi service are assigned to each task in the user request. Users can specify the type of services and local constraints like QoS preferences, global constraints, and other constraints like the total amount the user wishes to spend for the trip.

The system also captures the user's preferences over QoS parameters like frequency, reputation, cost, successful execution rate, and availability. QoS weights influence the ranking of web services. Also, after composition, the framework allows user to provide feedback which helps in evaluating the working of the system. Travel reservation system also allows service providers to register their web services.

### 4.2. QoS Aware Automatic Web Service Composition Framework

The core components of the QoS aware automatic web service composition (QAWSC) framework are service ranker and web service composer as is shown in Figure 3.

Web service discovery, QoS-based selection, and service ranker implement the user preference based web service ranking (UPWSR) algorithm. Web service composer which is the main crux of the proposed framework implements the QoS aware automatic web service composition (QAWSC) algorithm. Once the user submits the request UR(*T*, QWV, *C*), candidate web services for each task *t*_*i*_ in *T* are discovered from UDDI and ranked. Ranked services are used to generate composition plans. Composition plans are ranked and executed. The framework also captures user's feedback.

### 4.3. User Preference Based Web Service Ranking Algorithm

Web service providers register their web services to provide the service invocation parameters about the web services. For any service request raised by the web service requester, the candidate services are matched and retrieved from the service registry. The service request can be augmented with the user specific constraints on the QoS parameters. All the selected candidate services (satisfying the constraints) are then ranked using user preference based web service ranking (UPWSR) algorithm which is explained in Section 4.3.1. It mainly consists of web service discovery, QoS-based service selection, and service ranking.

#### 4.3.1. The Algorithm

The user preference based web service ranking (UPWSR) algorithm takes user request which consists of set of tasks *t*_*i*_ ∈ *T*, QoS weights, and set of web services WS_L_*i*__ that are registered in the service registry. Task *t*_*i*_ denotes the service type. For each task *t*_*i*_, list of ranked atomic services is returned by the algorithm (see Algorithm 1).

#### 4.3.2. Web Service Registration

Service providers register their web services and register the description of the web service in service registries like UDDI. Users access the Web Service Description Language (WSDL) document, which comprises the protocol bindings and message formats required to interact with the web services. Service providers publish the information about the functionality of the web service, providing details about the parameters that the service expects when it is invoked and other related information through the process of service registration. The registry has service ID and URI through which a web service can be accessed.

Nonfunctional aspects of the web services like average response time, cost, frequency, reputation, and so forth are stored in QoSDB. Suppose the service request contains “*n*” tasks (*t*_*i*_ to *t*_*n*_). First, the service type (functional aspect) required for each task in the service request is identified and stored. Service request also contains local constraints (QoS constraints) and global constraint. User preferences (QoS weight vector) over QoS properties and the constraints are stored. Service type and the list of web services WS_L_*i*__ are passed as input to the web service discovery component.

#### 4.3.3. Web Service Discovery

For each task in the service request, candidate web services are found using the web service discovery process. Web service discovery is the process of identifying and gaining access to the web services that matches with the functional requirement. Service registry is searched based on the “service type” required to complete each task. Search list (SL) or Service Provider List (SPL) contains the list of web services that satisfies the functionality required to complete each task.

Search list (SL) is given to the availability checker, to check whether the web service is available or not. Services that are not available are removed from the search list. Search list after removing the services that are not available is given to the QoS-based web service selection component. Services are accessed using service ID.

#### 4.3.4. QoS-Based Web Service Selection

QoS-based web service selection aims at finding best component services that meets the nonfunctional requirement like QoS. It calculates the average response time, frequency, success rate, reputation, and cost for each service in the search list. After calculating the QoS values, filtering is done. It compares all the QoS values of a service with other services and if a service is dominated by another service in all QoS parameters. For example, if service A has low cost, low response time, high frequency, high reputation, and higher success rate than service B, service B is eliminated. All the nondominated services are retained in the filtered list (FL).

Once the filtering operation eliminates the bad service providers, for each of the nondominated services, QoS parameter rank, that is, cost rank, reputation rank, frequency rank, success rate rank, and average response time rank, is calculated for each service. QoS-based ranked services are stored in the QoS ranked list (QRL).

#### 4.3.5. Service Ranker

A fuzzy ranking approach is employed by the service ranker to sort the services in the QoS ranked list based on the QoS criteria (cost, reputation, average response time, frequency, and success rate) and the QoS constraints (QoS weights specified by the user). Ranked services list (RSL_*i*_) contains the services for task *i* and these services are sorted based on the final rank.

The ranking of web services is based on Service Provider's Search Engine (SPSE) algorithm proposed by Zhao et al. [17]. The formula used to compute final rank for atomic services rank is described:

(5) Final  Ranki=CostRanki∗q1+SuccRateRanki∗q2+FreqRanki∗q3+RespRanki∗q4+RepRanki∗q5+AvailRanki∗q6,

where *i* denotes the position of web service in QoS ranked list and *i* varies from 1 to size of the QoS ranked list. *q*_1_ to *q*_6_ denote the QoS weight. After computing the final rank, the services are sorted based on the final rank and stored in a ranked services list (RSL).

Suppose there are *n* tasks required to complete the user request and ranked services list contains *m* candidate services for each task. So there can be *m* ^*n*^ compositions possible. To reduce the complexity and overhead involved in composition, Composition Influence Factor (CIF) is introduced in the approach. This factor limits the number of services for each task. This value can be specified by the user or the default value is used which determines the number of services in the ranked services list (RSL_*i*_) for each task. Hence, the number of possible compositions reduced from *m* ^*n*^ to (CIF)^*n*^ ranked services for each task is given to the web service composer.

### 4.4. QoS Aware Automatic Web Service Composition Algorithm

This section describes the QoS aware automatic web service composition (QAWSC) algorithm which takes the ranked services lists (RSL_*i*_) for each task in the user request and the constraints are taken as input. Web service composer generates composition plan from ranked services. Atomic services for each task in the user request are assigned and integrated.

Composition plan consists of service ID of the atomic web service that has been assigned to each task in the user request and execution pattern (serial pattern). QoS aware automatic web service composition (QAWSC) algorithm implemented by the web service composer is shown in Figure 4. Composition plan generator, aggregated QoS computation, constraint analyzer, Pareto optimal based selection, and user preference based ranking of composition plans are the major operations involved in web service composition. Ranked composition plans are executed and user can choose any of the composition plans.

#### 4.4.1. The Algorithm

User request which consists of tasks list, QoS weight vector, set of constraints, and ranked services lists for each task *t*_*i*_ in *T* are given as input to the web service composer which implements the QoS aware automatic web service composition (QAWSC) algorithm. Composition Influence Factor (CIF) determines the number of services in the ranked services lists for each task. First composition plans are computed from the ranked services and saved in the service composition table. Aggregated QoS values for all the generated composition plans are calculated. Composition plans that do not satisfy the constraints *C* specified by the user are eliminated. Then Pareto optimal based selection is used to select the dominant composition plans. Final rank is calculated using QoS weight vector and aggregated QoS rank. The ranked composition plan is executed. User's feedback is used to update the reputation score. QAWSC algorithm is explained as shown in Algorithm 2.

#### 4.4.2. Composition Plan Generator

Composition plan generator computes all possible composition plans from the ranked services list from the service ranker module. Cartesian product of the services in the list generates all possible combinations. The major steps in composition plan generator are

- creation of individual tasks tables,
- computation of service composition tables.

In the proposed travel reservation system, there can be three different tasks: travel, accommodation, and local transport reservation. QAWSC algorithm is implemented using the registry. Three separate tables named travel composition, hotel composition, and cab composition tables are created which are shown in Tables 2(a), 2(b), and 2(c).

As soon as the user submits the request, entries are deleted from those three tables. Based on the service type in the user request, services from the registry are added to these tables. Services that match with the service type are inserted into those tables. From the ranked services lists (RSL), based on the service type, services from the lists are entered into the corresponding tables. For example, if the service types in the service request are flight, Hotel_Deluxe, and taxi, then three lists (ranked flight service list, ranked Hotel_Deluxe service list, and ranked taxi services list) are created by the service ranker and inserted into the travel composition, hotel composition, and cab composition tables.

Suppose the ranked services list (RSL) contains “*m*” candidate ranked services for each task “*t*” and there are “*n*” tasks in the user request; possible compositions are *m* ^*n*^. Cartesian product of the ranked services list generates all possible service compositions. Join operation of travel composition, hotel composition, and cab composition tables; generate the possible composition plans and store them in the service composition table shown in Table 3. As soon as the user request is received by the travel reservation system, all the entries from the service composition table are deleted. Computed service compositions from the join operation of the individual tasks table are inserted.

#### 4.4.3. Aggregated QoS Computation

For all the composition plans in the service composition table, aggregated QoS values are calculated using Table 1. Composition plans are executed using serial execution pattern. Serial pattern is an execution pattern in which services are executed one after another and there is no overlap between execution periods of web services. Average response time of the composition plan is the sum of the average times required to complete a service request of its component services. It is the average of elapse times between request and response time of a web service. The reputation of the composition plan is the average ranking given by the end user according to their experiences. Reputation score given by the user ranges from 1 to 5. The frequency of the composition plan is the sum of the frequencies of the atomic services. It is the number of times the client used the web services. The cost of the composition plan is the sum of the execution costs of invoking atomic services. Successful execution rate of the composition plan is the average of the successful execution rates of the atomic service. After computing the aggregated QoS value of composition plans, it is stored in composition plan list (CPL) and given to constraint analyzer.

#### 4.4.4. Constraint Analyzer

Constraint analyzer is used to check all the composition plans, whether they satisfy the constraints specified by the user. It eliminates all the composition plans that do not satisfy the constraints.

Travel reservation system allows user to specify the budget range for the entire trip. Also the user can specify the constraints over the QoS. Aggregated QoS of composition plan should satisfy the constraints specified by the user. QoS properties can be classified as positive and negative QoS properties. QoS attributes like successful execution rate, reputation, frequency, and availability are positive QoS attributes. Higher the value of those positive QoS attributes; the efficiency of the composition process is high. Negative QoS attributes are average response time and execution cost. Lower the value of those negative QoS attributes; the efficiency of the composition is high. Equation (6) describes the constraint, where *i* denote the QoS property, CP denotes composition plan, and *C* denote the constraint specified by the user:

(6) $$\begin{array}{c} {\text{AggregatedQoS}}_{i}\text{ (CP) }\left\{\begin{array}{cc} \leq C_{i} & \left(\text{for negative QoS properties}\right)\\ \geq C_{i} & \left(\text{for Positive QoS properties}\right). \end{array}\right. \end{array}$$

Composition plan that satisfies the user constraints is saved in the Filtered Composition Plan (FCP) List and given to the Pareto optimal based selector.

#### 4.4.5. Pareto Optimal Based Selection

A Pareto optimal based selection is employed to delete the bad service composition plans in order to improve the efficiency of the web service composer. Based on the QoS values of the composition plans, if a composition plan is dominated by another composition plan in all QoS properties, then that plan is removed. Only compositions that are not dominated by other composition plans are retained. One thumb rule maintained by the Pareto optimal based selection is that the minimum response time composition plan, minimum execution cost composition plan, maximum frequency composition plan, maximum reputation composition plan, and maximum success ability rate composition plan are retained.

Pareto optimal based selection process reduces the complexity of the composition process by eliminating all the dominatable composition plans.  Table 4 shows the sample output of Pareto optimal based selection process. First the minimum response time composition plan, minimum execution cost composition plan, maximum frequency composition plan, maximum reputation composition plan, and maximum success ability rate composition plan are computed. Then elimination of dominating services is performed. Here composition plan CP_2_ is being dominated by CP_1_ in all QoS properties. Response time and cost are higher than CP_1_ and also frequency, successful execution rate, availability, and reputation of CP_2_ are lower than CP_1_. Hence CP_2_ is removed. Only the nondominated composition plans are retained in the Pareto optimal based selected list (POSL).

#### 4.4.6. User Preference Based Ranking on Composition Plans

Composition plans in the Pareto optimal based selected list (POSL) are sorted based on the average response time rank, cost rank, frequency rank, successful execution rate rank, availability rank, and reputation rank. Aggregated QoS ranks for all the composition plans in the Pareto optimal based selected list (POSL) are computed. For each composition plan, response time rank, cost rank, frequency rank, successful execution rate rank, availability rank, and reputation rank are stored as a structure as shown in Table 5.

After the aggregated QoS rank computation, QoS weight vector (QWV) specified by the user is multiplied by the corresponding QoS rank. Based on the user preference and QoS values, composition plans are sorted. Equation (7) shows the formula to calculate the final rank of composition plans:

(7) Final  RankCPi=CosRankCPi∗q1+SuccRateRankCPi∗q2+FreqRankCPi∗q3+RespRankCPi∗q4+RepRankCPi∗q5+AvailRankCPi∗q6.

Thus the proposed automatic web service composition supports flexibility in allowing the user to specify the preferences over composed services as well as individual web services. Composition plans are sorted based on the final rank and stored in the ranked composition plan list (RCPL).

#### 4.4.7. Feedback and Update

Ranked Composition plans are executed and the user can select any composition plan of his choice and view the response to the user's request. The user can select many composition plans from the list. QoS parameters like frequency, average response time, cost, successful execution rate, reputation, and availability of the composition plans can be viewed by the user. User provides feedback about the web services which improves the reputation score of that web service. Providing feedback is optional for the user. The user can click any of the composition plans from the ranked composition list. The user can view the details about the composed services. The user can provide the feedback by rating the service from 1 to 5, where 1 indicates that the service is poor, 2 denotes that the service is satisfactory, 3 indicates that the service is good, 4 indicates that service is very good, and 5 denotes that the service is excellent. As soon as the user provides feedback, reputation of that service is updated in the QoSDB which contains the QoS details of the web services.

## 5. Experimental Analysis

In this section, we present the results of our experiments to analyze the performance of QAWSC framework. Both the UPWSR and the QAWSC are analyzed. The performance measure is the execution time required by the proposed framework to satisfy the user request.

### 5.1. Experimental Setup

Our evaluation environment consists of three machines: QAWSC server (Intel Core i3 CPU, 2.13 GHz, 3 GB RAM, and Windows XP 3), which performs all the web service discovery, selection, ranking and composition; the client (Intel Core 2 Duo CPU, 2 GHz, 2 GB RAM, and Windows 7) which provides the user interface; the service registry (Intel Core i3 CPU, 2.13 GHz, 3 GB RAM, and Windows XP 3) to store the web services hosted by the web service providers along with the QoS related information, and, lastly, the composition plan repository to store the composition plans. We have utilized Java programming language to implement the UPWSR, QAWSC algorithms and all the machines used in the evaluation were in the same network.

Services in the registry are manually created. Services related to travel domain as shown in Table 6 are created. QoS information about those services is monitored regularly in QoSDB. Composition plans from the composition plan repository are deleted periodically. Service providers can register their services manually in the service registry and our proposed framework calculates QoS of those services dynamically.

### 5.2. Experimental Results

QoS parameters considered in our work are frequency, cost, reputation, response time, success rate, and availability. Here flight reservation, hotel of standard class, and renting the taxi are the set of tasks which are denoted as *t*_*i*_ and value of *i* ranges from 1 to 3. User preferences over the QoS parameters range from 1 to 6 where 6 denotes the highest value.

Let QoS weight vector QWV = 〈QWV〉 = 〈*qw*_1_, *qw*_2_,…, *qw*_*j*_〉, where *qw* denotes QoS weight specified by the user and *j* ranges from 1 to 6 indicating the corresponding QoS parameters. In this example value of *qw*_1_ is 3, value of *qw*_2_ is 4, value of *qw*_3_ is 3, value of *qw*_4_ is 4, value of *qw*_5_ is 5, and value of *qw*_6_ is 6. Budget lesser than Rs 20000 is the constraint specified by the user. The budget for the entire trip which includes flight booking, reserving a room in hotel of class standard, and renting a taxi should be lesser than Rs 20000. The experiments were carried out by increasing the number of services in the service registry. Services in the registry are increased from 100 to 500 with the step size of 100.

Figure 5 shows the performance of user preference based web service ranking (UPWSR) algorithm. Our UPWSR algorithm ranks the web services for each task and we have evaluated UPWSR algorithm for a single task and six QoS properties with user constraints over these parameters. Numbers of candidate web services are increased and time to rank those candidate web services also increases. QoS properties of the candidate web services are calculated dynamically, which increases the accuracy of the results.

Figure 6 depicts the performance of QoS aware automatic web service composition algorithm. Number of web services is increased from 100 to 500. Number of tasks in the user request is set to 3. Execution time for composition algorithm, that is, time taken to compose web services by the QAWSC, is the evaluation metric used. All the experiments repeated 10 times and average execution time is presented here.

Figure 7 depicts the performance of QoS aware automatic web service composition framework by increasing the number of tasks. Number of web services is increased from 100 to 500 and number of tasks in the user request is set to 3, 5, and 10. Number of candidate services for each task is also increased. Execution time for composition algorithm, that is, time taken to compose web services by the QAWSC, is the evaluation metric used. All the experiments repeated 10 times and average execution time is presented here.

*Working Example*. For the web service “Ginger Hotels,” the three operations identified from the WSDL are bookRoom, getAvailability, and getBookingHistory as given in Figure 8. A sample set of data is obtained from the service provider and based on the numerous other clients that are created. A certificate is issued to the web service based on the values obtained in the quality assessment phase as specified in Figure 9. The certificate along with the WSDL document is then registered to the jUDDI, the service registry.

Any service request raised is parsed syntactically and semantically to identify the keywords. For example, for a query for “*Travel from Chennai to Salem*,” the keywords obtained are travel, mode-of-transport, taxi, hotel, tourist-interest, and so forth. The keyword “travel” derives from the service request; the result is obtained by matching “travel” with domain ontology and retrieving the related concepts. The service selection algorithm uses the keywords and conditions the presence of functional and nonfunctional properties of the web services and the QoS requirements of the service request. The services are ranked based on the parametric data available on the certificate (issued by the QoS agent). The composition plans are generated by configuring an action plan, eliminating the faults, negotiation, and ranking of compositions as shown in Figure 10.

From the available set of 6 services (in our example), five compositions could be derived. However, availability of a candidate web service influences the availability of the composition. The best available composition is composition 1 as shown in Table 7. Even though the availability is increased with composition 5, there exists incompatibility between Services C and F and hence it is not considered in Table 8.

Table 8 is the interface provided to the web service requester as the result of invoking the proposed QBroker Framework. Providing the top *n* web service compositions to the service request makes the framework more reliable. On selection of an option in the plan offered, a BPEL file is created and the web service composition is executed and provided to the service requester for further usage. The composition is also saved for future reference and undergoes a feedback analysis to utter impressive composition delivery.

The time taken by the UPWSR algorithm to rank the candidate web services for each task increases by very small duration with the increase in the number of web services in the service registry. It mainly depends on the number of candidate web services. Computation time of QAWSC algorithm increases linearly with the increase in number of web services. Computation time of QAWSC algorithm mainly depends on the number of services in the ranked services list (RSL). By changing the number of the services in ranked lists, computation time of QAWSC algorithm can be significantly reduced. Composition Influence Factor decides the number of the services in the ranked services lists. We set the value of CIF to 100. This factor should be set manually before any user sends the request. CIF is used to reduce the complexity of the QAWSC algorithm. Number of possible composition reduced from *m* ^*n*^ to (CIF)^*n*^, where *m* denotes number of ranked services and *n* denotes the number of tasks in the user request.

## 6. Conclusion

The proposed framework addresses the challenge issues web service composition. We proposed a QoS aware automatic web service composition framework which is flexible in satisfying multiple QoS requirements and also considers the user preferences. We proposed a user preference based ranking algorithm which reduces the overhead in web service composition. User can specify his preferences over QoS parameters which makes the web service composition more flexible. The proposed approach dynamically composes web services and the composition plans are generated automatically. We have considered six QoS criteria and also considered user's constraints over these parameters. Our system also allows user to provide feedback after composition which updates the reputation of those services immediately. We have evaluated our algorithm based on the computation time for ranking and composition based on different number of service providers and number of tasks. Our experiments showed that our QAWSC composition framework yields lower execution time and supports user preferences. We have implemented our framework for travel application. In the future, we plan to test our framework using standard datasets like WS-Challenge datasets.

## Figures and Tables

**Figure 1:** Web service architecture.

**Figure 2:** Travel reservation scenario.

**Figure 3:** QoS aware automatic web service composition framework with UPWSR.

**Figure 4:** QoS aware automatic web service composition framework.

**Figure 5:** Performance of UPWSR.

**Figure 6:** Performance of QAWSC.

**Figure 7:** Performance of QAWSC for different number of tasks.

**Figure 8:** Service registration.

**Figure 9:** QoS assessment for web service: Ginger Hotels.

**Figure 10:** Composition generated for the service request.

**Algorithm 1:** User preference based web service ranking algorithm (UR(*T*, QWV, *C*), WS_L_*i*__).

**Algorithm 2:** QoS aware web service composition algorithm (UR(*T*, QWV, *C*), RSL_*i*_).

**Table 1:** QoS aggregation function.

Sl. number	QoS criteria	Sequence
1	Execution cost (CP_*i*,*C*_)	∑_*i*=1_^*n*^ *C*(WS_*i*_)
2	Successful execution rate (CP_*i*,*S*_)	(∑_*i*=1_^*n*^ *S*(WS_*i*_))/*n*
3	Response time (CP_*i*,*T*_)	∑_*i*=1_^*n*^ *T*(WS_*i*_)
4	Reputation (CP_*i*,*R*_)	(∑_*i*=1_^*n*^Rep(WS_*i*_))/*n*
5	Frequency (CP_*i*,*F*_)	∑_*i*=1_^*n*^ *F*(WS_*i*_)
6	Availability (CP_*i*,*A*_)	∏_*i*=1_^*n*^ *A*(WS_*i*_)

**(a):** 

Service ID	Source	Destination	Mode	Amount
11	Chennai	Goa	Flight	15000
100	Chennai	Kolkata	Train	3000
21	Chennai	Delhi	Flight	20000
45	Chennai	Bangalore	Bus	1000
300	Bangalore	Chennai	Flight	7500

**(b):** 

Service ID	Destination	Class	Amount
101	Goa	Hotel_Standard	2000
10	Kolkata	Hotel_Deluxe	3000
210	Delhi	Hotel_Economy	500
50	Bangalore	Hotel_Standard	1000
30	Chennai	Hotel_Standard	750
122	Goa	Hotel_Economy	400
134	Kolkata	Hotel_Economy	450
201	Delhi	Hotel_Deluxe	3000

**(c):** 

Service ID	Destination	Type	Amount
75	Goa	Taxi	200
11	Kolkata	Jeep	300
21	Delhi	Van	500
5	Bangalore	Taxi	100
3	Chennai	Taxi	75

**Table 3:** Service composition table.

Composition ID	Travel_ID	Travel_Name	Hotel_ID	Hotel_Name	Cab_ID	Cab_Name
1	11	Flight Service H	101	Hotel Service A	201	Van Service A
2	11	Flight Service H	101	Hotel Service A	202	Van Service B
3	11	Flight Service H	101	Hotel Service A	203	Van Service C
4	11	Flight Service H	101	Hotel Service A	204	Van Service D
5	11	Flight Service H	101	Hotel Service A	205	Van Service E

**Table 4:** Example of Pareto optimal based selection.

Composition plan ID	Response time (ms)	Cost (Rs)	Frequency	Succ. rate (%)	Reputation (1 to 5)	Availability
CP_1_	400	500	590	78	4	0.6
CP_2_	500	700	56	43	1	0.75
CP_5_	678	765	567	65	2	0.8

**Table 5:** Aggregated QoS rank example.

Composition plan ID	Response time rank	Cost rank	Frequency rank	Succ. rate rank	Reputation rank	Availability rank
CP_12_	4	5	59	8	4	6
CP_2_	5	7	56	3	1	5
CP_5_	8	65	7	65	2	8

**Table 6:** List of web services.

S. number	Functionality of the web service	Web service types
1	Travel services	Flight/train/bus
2	Accommodation services	Hotel deluxe/hotel standard/hotel economy
3	Local transport rental services	Jeep/van/taxi

**Table 7:** Possible compositions from the available web services.

Compositions	Web services	Availability
1	A-C-E	73
2	B-C-E	72
3	B-D-F	71
4	B-E-F	71
5	A-C-F	83

**Table 8:** Generated composition plans.

Plan	Rank	Action
SouthernrailwaysSR12054ChennaiToSalem GingerhotelsSalem HelitaxiSalem	1	

KsrtcKSRTC12036ChennaiToSalem GingerhotelsSalem HelitaxiSalem	2	

KsrtcKSRTC12036ChennaiToSalem GingerhotelsSalem InfotaxiSalem	3	

KsrtcKSRTC12036ChennaiToSalem RamhotelsSalem InfotaxiSalem	4	
